# Assessing the asymmetric impact of physical infrastructure and trade openness on ecological footprint: An empirical evidence from Pakistan

**DOI:** 10.1371/journal.pone.0262782

**Published:** 2022-05-17

**Authors:** Samia Zahra, Dilawar Khan, Rakesh Gupta, József Popp, Judit Oláh

**Affiliations:** 1 Higher Education Archives and Libraries Department, Khyber Pakhtunkhwa, Pakistan; 2 Kohat University of Science and Technology, Kohat, Pakistan; 3 Department of Accounting, Finance and Economics, Griffith University Brisbane, Brisbane, Australia; 4 Department of Management, Faculty of Applied Sciences, WSB University, Dabrowa Górnicza, Poland; 5 Faculty of Economics and Business, University of Debrecen, Debrecen, Hungary; 6 College of Business and Economics, University of Johannesburg, Johannesburg, South Africa; Universiti Malaysia Sabah, MALAYSIA

## Abstract

This study analyzed the asymmetric impact of the physical infrastructure and trade openness on Pakistan’s ecological footprint over the period 1970–2019 using the non-linear autoregressive distributed lag model. The study results posit that positive and negative shocks to physical infrastructure increase and decrease the ecological footprint asymmetrically in the short-run and symmetrically in the long-run. Likewise, the positive and negative shocks to trade openness increase and decrease the ecological footprint asymmetrically, both in the short and in the long run. Furthermore, urbanization also positively and significantly increases Pakistan’s ecological footprint in the short and long run. Moreover, a 1% increase in physical infrastructure increases the ecological footprint by 0.32%, while a 1% decrease in physical infrastructure decreases the ecological footprint by 0.33% in the long run. Similarly, a 1% increase in trade openness causes a 0.09% increase in the ecological footprint in the long term, while a 1% reduction in trade openness causes a 0.61% reduction in the ecological footprint. The results also conclude that urbanization is a major determinant of Pakistan’s long-term ecological footprint. Thus, a 1% increase in urbanization causes a 1.31% increase in the ecological footprint in the long run. Finally, this study recommends that policies regarding physical infrastructure be formulated keeping in view its environmental impact. In addition, strict environmental policies should be implemented to reduce the environmental degradation effect of trade openness.

## Introduction

Ecological footprint theory seeks is to determine the amount of land required to supply food, water, fuel, and shelter or human exploitation of the ecosystem to meet needs. The best way to estimate an individual’s ecological footprint is to calculate how much area is used by their life or all land for living purposes. The ecological footprint combines the two concepts to address the damage that human activity causes at the ground level and the damage from the use of all the Earth’s natural resources that are not returned. Human activities endanger the environment and ecosystem, which provide food, clean water, electricity, recreation, and green space. The usage of Earth’s resources by humans has exceeded bio-capacity. As a conclusion, humanity will require the regeneration capacity of 1.6 Earths to meet its ecological service needs. Development indicators has already outstripped the planet’s ability to provide it, resulting in an ecological deficit in many countries. Around 80% of the world’s population lives in a country with a serious environmental problem. Nations must observe their ecological constraints to ensure sustainable development [1]. Human living standards and well-being have risen dramatically in recent decades because of significant economic expansion and prosperity [2]. However, this growth has degraded environmental quality because it depends mainly on human demand for water, infrastructure, energy, and food, among other things, resulting in emissions, loss of biodiversity and environmental imbalance [3–5]. Environmental pressure is created by human demand for water, infrastructure, energy, and food, among other things, resulting in emissions, loss of biodiversity and environmental imbalance [3–6]. While the contribution given to environmental protection was deemed to be the most important environmental component of bioenergy projects [7]. Alola, Bekun [8] and Qin [9] suggest that human exploitation of commodities and ecosystem services is a cause of modern concerns about environmental destruction, global warming, ecological imbalances, and economic failures.

Global economic activity has exacerbated the problems of environmental deterioration and pollution. Industrial development, growing urbanization, and modern farming practices are among the activities [10]. Increase in pollution results from productivity expansion and economic growth has a detrimental impact on environmental deterioration and climate change [11]. Because it covers built-up land, CO_2_ emissions, agricultural land, fisheries, pastures, and forest products [1], the ecological footprint is a more comprehensive assessment or measure than the CO_2_ emission which is formerly employed as an environmental proxy most of the time [12, 13]. The ecological footprint method is being used to estimate the overall human burden on natural ecosystems as a first approximation (Lin et al., 2015; Lin et al., 2018; Ghiţă [14]; Ullah & Khan, 2020), but with some recognized disadvantages [15, 16]. Many factors must be considered to assess the impact that individuals have on the environment, one of which is indirect and caused by their actions. Individual impact on the environment includes developing renewable resources, dealing with urban growth and expansion, accommodating a growing population and road networks, and recycling or transporting waste, increasing the magnitude of the footprint. With the development of human activity, directly or indirectly, more emphasis has been given to the environmental consequences of population density, energy consumption, economic expansion, trade policy, and other noteworthy elements [8, 17–23].

Infrastructure investment is a critical determinant of economic growth and development [24, 25]. Using various econometric methodologies and samples, several studies empirically investigated the favorable influence of infrastructure investment on output production and growth [26–28]. However, it has a detrimental impact on environmental sustainability [29, 30]. It is estimated that physical infrastructure, such as power plants, concrete roads, bridges, mines, oil refineries, mines and waste factories, create a considerable amount of environmental deterioration [31]. In the era of industrialization, the transport sector and investment in transport infrastructure are considered the main determinants of environmental deterioration [29, 32–42].

Rapid urbanization has also led to lifestyle changes and, as a result, population in cities has expanded dramatically in recent decades [43–45]. The urbanization process is one of economic and social renovation and transformation. It is the migration of people from rural areas to urban cities and metropolitan and the methodical shift from an agrarian to an industrial sector [46]. The immediate effects of urbanization include visible changes in land consumption [47], but there are also indirect and intertwined effects [48]. The world has seen tremendous urbanization in recent decades, the global urban population has grown from 751 million in 1950 to 4.2 billion in [49]. In addition, it is expected to reach 6.4 billion over the next 30 years [46]. To support this extraordinary expansion, the new urban infrastructure requires accommodation of the urban population, thus increasing the per capita ecological footprint. While urbanization is a factor responsible for increasing environmental degradation [50]. While Increase in land use may result in the destruction of agricultural land and its systems, resulting in widespread devastation [51].

The degree of income determines the inflow of FDI and, in turn, commercial openness. However, the effect of trade openness and FDI on the environment is controversial. According to the “pollution haven effect”, As a result of insufficient environmental regulation, low-income countries attract more FDI, resulting in increased pollution. Contrary, Dinda [52] states that FDI and trade openness can reduce pollution in low-income nations by stimulating the economy, creating jobs, increasing income levels, and facilitating knowledge transfer, a phenomenon known as " pollution halo effect ".

Pakistan is the world’s most vulnerable country to climate change, since environmental issues have become a top priority for Pakistan’s government, as well as for other developing nations [2, 53]. In the previous 20 years, Pakistan has been one of the ten most vulnerable regions to climate change. Energy and transportation are the most polluting sectors, accounting for half of all pollution [53]. Carbon emissions are currently increasing by 6% per year and will reach 400 Mt CO_2_ equivalent (per year) by 2030 in Pakistan if current trends continue (World Bank, 2019), which is an alarming increase. In addition, between 1999 and 2018, Pakistan lost 0.53 percent of its GDP and sustained economic losses of roughly US$3,792.53 million as a result of 152 extreme weather events [54].

This study adds to the previous literature in several ways. First, most previous studies have analyzed the symmetrical association between trade and the environment, using variables such as trade openness or total trade in environmental emissions and the impact of physical infrastructure on environmental degradation, although this is the first study to explore the asymmetric impact of trade openness and physical infrastructure on the ecological footprint in Pakistan. This study fills the existing gap, using non-linear ARDL. Second, a physical infrastructure index was developed using the principal component analysis (PCA) technique to include the important physical infrastructure components. Finally, most previous studies have used carbon dioxide (CO_2_) emissions as a proxy to capture environmental degradation; this study used the ecological footprint as a proxy for environmental quality. Therefore, the ecological footprint measured in global hectares (gha) is the best proxy for environmental quality compared to carbon dioxide (CO_2_) emissions [8, 13, 17, 18, 21, 44, 55–63].

In addition, environmentalists, policymakers and government officials will benefit from the study’s findings. This study provides a deeper understanding and information environmental protection. The rest of the article is briefly discussed below. The literature review directly or indirectly related to this study is explained in the “Literature Review” section. The data, model and methodology were explained in the section entitled "Research Methodology". The study results and their interpretation are presented in the "Results and Discussion" section. Finally, conclusions and policy implications based on the study’s findings are provided in the "Conclusions and Policy Implications" section.

## Literature review

Several studies have been undertaken in the past to investigate the symmetric influence of physical infrastructure, trade openness, and urbanization as significant environmental degradation factors. Zhi-Guo, Cheng [64] suggests that various economic sectors increase carbon emissions, and academics have highlighted which areas are most significant for institutions and governments, which need immediate attention. Accompanying the growth of industrialization and urbanization, the transportation has a significant and progressive or positive impact on global carbon emissions [53, 65]. Timilsina and Shrestha [38] investigated different determinants of emission in transport sector over the period 1980 to 2005 for selected Asian countries. It is concluded that per capita income, population and increasing trends in transport ultimately lead to increased CO_2_ and therefore cause environmental degradation. Similarly [66, 67], empirically investigated that growth in transport sector to increase in CO_2_ and environmental pollution. Baabou, Grunewald [48] investigated significant determinants of the ecological footprint in Mediterranean cities and concluded that, in addition to different factors such as an increase in food intake and manufactured commodities, other socioeconomic factors such as transport, physical infrastructure and increased disposable income and changes in cultural trends are important factors of the ecological footprint.

However, Moore, Kissinger [68]; Sierra, Flores [69]; Wackernagel and Rees [61] suggest that proper management in the physical infrastructure and transportation sector can benefit economic growth. They suggested that vehicle mileage taxes provide direct and indirect benefits at many scales, such as reducing pollution, improving air quality, promoting public safety and health, and reducing fossil fuel consumption and increasing employment in public transportation. Due to the proximity of many different activities, urban environments also provide the potential for economies of scale. Gassner, Lederer [70] investigated the ecological footprint of public transport (a driver of physical infrastructure) in Vienna, Austria, and concluded that transport and its accessories contribute to ecological carbon emissions. Some studies have also concluded that an increase in population and increased returns on urbanization and transport lead to increased land use, carbon emissions and consumption of land resources. Therefore, these factors are the main determinants of the increase in the per capita ecological footprint [55, 56, 61, 68, 71]. As a result, not only do transportation and related infrastructure raise CO_2_ emissions and environmental deterioration, but they also increase land consumption. This land usage is not even evenly distributed among the various modes of transportation infrastructure, resulting in its dominance as a driver of the ecological footprint in various capacities [70]. Several studies, such as [56, 70, 72–77] assessed the contribution of the public transport network, partial transport infrastructure, land use for transport in the context of the carbon footprint with respect to overall life cycle emission and environmental degradation.

Considering the ecological footprint as the most reliable measure of the environment and its quality, Nathaniel [43] the impact of urbanization, trade, and economic expansion on ecological footprint of Indonesia was explored. The study finds that economic growth and urbanization significantly increase environmental degradation. Trade is a short-term determinant of ecological footprint and environmental quality, while long-term factors of ecological footprint and environmental quality are energy use urbanization, and economic growth. Nathaniel, Nwodo [45] empirically investigated the impact of urbanization and trade on the ecological footprint in CIVETS over the period 1990 to 2014. By employing the AMG technique, the study concluded that trade is a positive and significant determinant of environmental quality, while urbanization is a negative, but significant factor of environmental quality. Likewise, Kurniawan and Managi [78] investigated the impact of urbanization and trade on fossil fuel (coal) consumption from 1970 to 2015, and both variables multiply coal consumption, which has a detrimental impact on environmental degradation. The study suggested a decrease in coal depletion in Indonesia to achieve environmental goals. Alola, Bekun [8] also empirically investigated that trade, fertility, and energy have all had an impact on Europe’s ecological footprint between 1997 and 2014. The study concluded that trade and fertility deteriorate environmental sustainability. The study concludes that trade and fertility deteriorate environmental sustainability. Dogan, Taspinar [59] explored the key drivers and determinants of ecological footprint in MINT countries from 1971 to 2013. The study investigated that exports, increased energy consumption, and urbanization are the significant factors or drivers responsible for ecological pressure in MINT countries. Ulucak and Khan [79] found that Environmental Curve Kuznets is valid in each of the BRICS countries. The study also explored the determinants for decreasing the ecological footprint in the mentioned countries, using the empirical methods DOLS and FMOLS for the period 1992 to 2016. In the BRICS countries, urbanization was discovered to be a negative factor of the ecological footprint. On the contrary, Ahmed, Zafar [62] found urbanization as positive and significant determinant of ecological footprint in G7. Likewise, Ahmed, Asghar [80] investigated the influence of urbanization, economic growth and natural resources on China’s ecological footprint and found urbanization and growth as positive determinant of ecological footprint. Baloch, Zhang [81] investigated for the period 1990 to 2016, the influence of financial development, GDP, FDI, and urbanization on the ecological footprint of 59 Belt and Road countries. All these variables were found to be positive drivers of environmental deterioration and ecological footprint in the nations studied.

Regardless of the previous literature, the new study fills a research gap in a variety of ways. To begin with, previous empirical studies have looked at the linear or symmetric relationship between physical infrastructure and environmental degradation, whereas this is the first study to look at the asymmetric impact of physical infrastructure on environmental degradation using a more comprehensive environmental proxy, the ecological footprint. Secondly, physical infrastructure index is developed through PCA approach by including important components of physical infrastructure in Pakistan.

## Methodology

The core objective of this study was to investigate the asymmetric impact of physical infrastructure and trade openness on the ecological footprint in Pakistan for over the period 1970–2019. An index was developed for the physical infrastructure in Pakistan using the Principal Component Analysis (PCA) approach. Although there are many techniques used to interpret large datasets, PCA is most widely used because it reduces the dimensionality of the data in a comprehensible manner and preserves most of the data information intact [82]. Second, it also accumulates data while eliminating the autocorrelation problem [83]. The infrastructure index was calculated including five physical infrastructure components. These include the length of roads measured in thousand kilometers (000 Kms.), rail route measured in thousand kilometers (000 Kms.), mobile phone subscription measured in thousands of numbers (000 Nos.), landline subscription measured in thousand numbers (000 Nos.), and the route of Pakistan International Airlines (PIA) measured in thousand kilometers (000 Kms.) [84]. The prime measure of trade openness is the trade intensity ratio and is referred to as export plus import divided by GDP. In addition, urbanization was measured as the urban population measured in thousand people (000 people) [85].

The ecological footprint (EF) measured in global hectare (gha) was taken is taken as dependent variable. As the ecological footprint covers built-up land, CO_2_ emissions, agricultural land, fishery regions, grazing land, and forest products, it is a more comprehensive estimate than the previously used CO_2_ emission as an environmental indicator [1]. Physical infrastructure measured as infrastructure index (II) and trade openness (TO) [85] were used as independent variables. Physical infrastructure is a significant determinant of environmental degradation [53] Improvement in physical infrastructure give way to an increase in economic growth, ultimately paving the way for an ecological footprint [2]. Likewise, trade openness is also considered an important factor in the deterioration of environmental quality [86, 87]. Urbanization (UR) measured as urban population per thousand people [85] was also included as an independent variable to avoid model specification errors. Moreover, urbanization is also considered a significant factor in environmental contamination, in view of the previous literature. As a result of rampant urbanization, ecological degradation is happening very quickly, causing many problems such as property insecurity, water contamination, excessive air pollution, noise, and garbage disposal issues are need to be addressed [88]. It also causes congestion in cities and large population requires more jobs and other requirements. These factors increase economic activities, including the expansion of industrial zones, heavy traffic, higher levels of various pollutions [5]. The description and sources of the data series are explained in Table 1.

**Table 1:** Description and sources of the data series.

Abbreviation	Description		Data source
EP	Ecological footprint measured in thousand global hectares (gha)		Global Footprint Network (2021)
II	Physical infrastructure Index		
	This index was computed including the following components:		
	1) Rd	Length of roads (measured in thousand Kms.).	Pakistan Economic Survey (2020)
	2) Rr	Rail route (measured in thousand Kms.).	Pakistan Economic Survey (2020)
	3) Ms	Mobile phone subscription (measured in thousand Nos.).	Pakistan Economic Survey (2020)
	4) Ls	Landline subscription (measured in thousand Nos.).	Pakistan Economic Survey (2020)
	5) Ar	Airline route (measured in thousand Kms.).	Pakistan Economic Survey (2020)
TO	Trade openness measured as export plus import divided by GDP.		World Bank (2020)
UR	Urban population (measured in thousand people).		World Bank (2020)

First, it is important to determine the stationarity of time series data to avoid spurious results. According to Granger and Newbold [89] the application of standard OLS techniques to unit root data leads to spurious regression. Autoregressive of order one AR(1) model is used to investigate the stationarity condition which is given below:

$$Z_{t}=£\;Z_{t-1}+\in_{t}$$ (1)

The behavior of the time series of *Z*_*t*_ depends on its previous value *Z*_*t*−1_ is an axiom of the AR (1) model. There may be three possible instances of this model below:

If|£|<1;stationaryseries.

If|£|>1;explosiveseries.

If|£|=1;non‐stationaryseries.

This study applied the Augmented Dickey-Fuller (ADF) test [90] and the Phillips Perron test [91] to verify stationarity in data from this time series. The Akaike Information Criteria (AIC) is a criterion for determining the best lag time. These two equations from the ADF test were utilized to predict the non-stationarity problem mathematically.


$$\Delta Z_{t}=\alpha_{0}+£\;Z_{t-1}+\sum_{i=1}^{n}\beta_{i}\Delta Z_{t-1}+\in_{t}$$ (2)

$$\Delta Z_{t}=\alpha_{0}+\alpha_{1}Z+£\;Z_{t-1}+\sum_{i=1}^{n}\beta_{i}\Delta Z_{t-1}+\in_{t}$$ (3)

*α*_0_ denotes the term intercept while £ exhibits the trend variable co-efficient. ∈_*t*_ is used for the error term at time *t* in the selected model. For the Augmented Dickey Fuller test, null hypothesis assumes that the data are not stationary.

The PP test is also used to investigate the stationarity problem in the data determined by the two equations below:

$$\Delta Z=\alpha_{0}+£\;Z_{t-1}+\xi_{t}$$ (4)

*α*_0_ is intercept symbol, £ is co-efficient of slope, *β*_1_ is trend variable coefficient and *ξ*_*t*_ is time *t* residual.

Second, this study applied nonlinear auto-regressive distributed lag (NARDL) model [92] to examine the asymmetric impact of physical infrastructure and trade openness on Pakistan’s ecological footprint. The impact of the ecological footprint (EP) on physical infrastructure (II), trade openness (TO), and urbanization (UR) is expressed using the following mathematical specification:

$$EP_{t}=\alpha_{0}+\alpha_{1}II_{t}+\alpha_{2}TO_{t}+\alpha_{3}UR_{t}+\varepsilon_{t}$$ (5)

Where *α*_0_, *α*_2_, *α*_3_ show the model parameters, and *ε*_*t*_ is the normally distributed residual term with mean is equal to zero and constant variance.

The empirical specification of this study starts from the usual symmetric ARDL model proposed by [93]. Therefore, the auto-regressive distributed lag (ARDL) model is written as under:

$$\Delta \log EP_{t}=\alpha_{0}+\sum_{k=1}^{m}\alpha_{1i}\Delta \log EP_{t-k}+\sum_{k=0}^{m}\alpha_{2i}\Delta \log II_{t-k}+\sum_{k=0}^{m}\alpha_{3j}\Delta \log TO_{t-k}+\sum_{k=0}^{m}\alpha_{4k}\Delta \log UR_{t-k}+\beta_{1}log{EP}_{t-1}+\beta_{2}\log II_{t-1}+\beta_{3}\log TO_{t-1}+\beta_{4}{logUR}_{t-1}+\varepsilon_{t}$$ (6)

In Eq (6), *α*_*i*_ and *β*_*i*_ show long run and short-run coefficients, respectively, while Δ shows the difference operator for unit root; ∈_*t*_ represents the residual term with mean is equal to zero and constant variance.

Following [92] through the asymmetric modification in linear long-run and short-run empirical analysis *II*_*t*_, *TO*_*t*_ are decomposed into the partial sum of two new time series variables for each of the variables. More specifically, one determines the positive partial sum of positive changes in the physical infrastructure and trade openness which is ${II}_{t}^{+}{TO}_{t}^{+}$ and the other is ${II}_{t}^{-},\;{TO}_{t}^{-}$ as the partial sum of negative fluctuations in the physical infrastructure and Trade openness. Because the negative asymmetric variable is missing, the urbanization variable cannot be turned into an asymmetric variable [94]. The specification is given below in Eq 7, 8, 9, 10.


$$II_{t}^{+}=\sum_{m=1}^{t}II_{t}^{+}=\sum_{m=1}^{t}\max(\Delta II_{t}^{+},0)$$ (7)

$$II_{t}^{-}=\sum_{m=1}^{t}\Delta II_{t}^{-}=\sum_{m=1}^{t}\min(\Delta II_{t}^{-},0)$$ (8)

$$TO_{t}^{+}=\sum_{m=1}^{t}TO_{t}^{+}=\sum_{m=1}^{t}\max(\Delta TO_{t}^{+},0)$$ (9)

$$TO_{t}^{-}=\sum_{m=1}^{t}\Delta TO_{t}^{-}=\sum_{m=1}^{t}\min(\Delta TO_{t}^{-},0)$$ (10)

Eq (11) inserts the partial sum of the positive and negative fluctuations of *II*_*t*_ and *TO*_*t*_ as (${{II}_{t}^{+},TO}_{t}^{+}$), and (${{II}_{t}^{-},TO}_{t}^{-}$) to examine the short run and long run asymmetric of physical infrastructure and trade openness on ecological footprint in Pakistan is given as follows:

$$\Delta \log EP_{t}=\alpha_{0}+\sum_{k=1}^{m}\alpha_{1i}\Delta \log EP_{t-k}+\sum_{k=0}^{m}\alpha_{2k}\Delta \log II_{t-k}^{+}+\sum_{k=0}^{m}\alpha_{3k}\Delta \log II_{t-k}^{-}+\sum_{k=0}^{m}\alpha_{4j}\Delta \log TO_{t-k}^{+}+\sum_{k=0}^{m}\alpha_{5j}\Delta \log TO_{t-k}^{-}+\sum_{k=0}^{m}\alpha_{6j}\Delta \log UR_{t-k}+\beta_{1}\log II_{t-k}^{+}+\beta_{2}\log II_{t-k}^{-}+\beta_{3}\log TO_{t-1}^{+}+\beta_{4}\log TO_{t-1}^{-}+\beta_{5}\log UR_{t-1}+\varepsilon_{t}$$ (11)

Eq (11) calculates the asymmetric or non-linear influence of physical infrastructure index and trade openness on Pakistan’s ecological footprint in the short and long run, considering the short- run and long-run partial sum of positive and negative variations of the model. Furthermore, the Wald test was utilized to establish the asymmetric short-run and long-run effects of Pakistan’s physical infrastructure index and trade openness on the ecological footprint. It is important to remember that lag order selection can help to figure out the best delay period for non-linear ARDL model. To identify the most appropriate lag length, various selection measures are applied. The best lag length of the model is determined using AIC as a standard measure or criteria in this study.

Finally, appropriate diagnostic tests are used to determine the reliability, stability, and predictability of NARDL coefficients of the model. The Breusch -Godfrey LM test [95, 96] was used to verify the residuals auto-correlation and serial correlation. The Jarque-Bera test and the Ramsey’s RESET test (Ramsey, 1969) were used to verify the normal distribution of the residual terms and the appropriate functional form of the model. In addition, CUSUM (cumulative sum of residuals) and CUSUMQ (cumulative sum of squared residuals) tests were used to verify the stability of the non-linear ARDL parameters [97].

## Results and discussion

This paper explored the asymmetric impact of physical infrastructure and trade openness on Pakistan’s ecological footprint. First, the physical infrastructure index was developed using the Principal Component Analysis (PCA) approach. This approach is most widely used because it reduces the dimensionality of the data in a comprehensible manner and preserves most of the data information intact [82]. Furthermore, it also accumulates data while eliminating the autocorrelation problem [83]. The physical infrastructure index was computed including five physical infrastructure components. These include the road length measured in thousand kilometers (000 Kms.), Rail route measured in thousand kilometers (000 Kms.), Mobile phone subscription measured in thousands of numbers (000 Nos.), Landline subscription measured in thousand numbers (000 Nos), and the route of Pakistan International Airlines (PIA) measured in thousand kilometers (000 Kms.) (Pakistan Economic Survey, 2020). The Results of the physical infrastructure index aggregation are given in Table 2. The first panel of the table shows the correlation between the components of the physical infrastructure index. The road length with rail route; rail route with mobile subscription, landline subscription, airline route; mobile subscription and airline route pair, have a negative correlation. Likewise, the road length with mobile subscription, landline subscription and airline route; mobile subscription with landline subscription; and landline subscription with airline route, have a negative correlation. Moreover, Table 2 shows that there are weak and strong autocorrelations between the variables, implying that the parameters would be misleading and spurious in the estimate if all five determinants of physical infrastructure were included in a single regression. In addition to causing misleading and spurious regression, the information in this example is more representative and sufficient than a single indicator would have discovered. The second penal in the table shows specific deviation by PCA components which shows that the first to the fifth component has explanatory powers ranging from 52.97% to 1.42% which shows that the first component has variations of 52.97% in the physical infrastructure index. It is concluded that, when compared to other components of the infrastructure index, the first component has the greatest explanatory power to better account for variations in physical infrastructure. It is vital to consider that the estimates shown in the fifth column are used to quantify the final physical infrastructure index depth indicator provided in the subsequent regression.

**Table 2:** Physical infrastructure index aggregation.

Variables	Road length	Rail route	Mobile subscription	Landline subscription	Airline route
Correlation Matrix					
Road length	1.0				
Rail route	-0.23	1.0			
Mobile subscription	0.63	-0.12	1.0		
Landline subscription	0.89	-0.19	0.62	1.0	
Airline route	0.51	-0.18	-0.17	0.37	1.0
Component Analysis					
Components	Eigen Values	% Variance	Cumulative Proportion %	First Principal Component	
1	2.65	52.97	52.97	(0.59)^Rd^	
2	1.20	23.90	76.87	(-0.21)^Rr^	
3	0.90	17.91	94.78	(0.43)^Ms^	
4	0.19	3.80	98.58	(0.57)^Ls^	
5	0.07	1.42	100.0	(0.29)^Ar^	

Note. The numbers in parentheses are estimated coefficient values for the respective superscript variable.

Table 3 displays descriptive statistics of the data series. Descriptive statistics helps to understand the basic characteristics and trends of the data series. The average value of the ecological footprint is 50674.6 thousand global hectares (gha) with a median 50920.5, ranging from 30101.5 to 68301.3. Likewise, the average value of physical infrastructure index, trade openness, and urban population have average values of 4.0, 0.36 and 41576.9 thousand people with a median of 4.2, 0.35 and 38709.3, respectively.

**Table 3:** Descriptive statistics of the data series.

Variables	Mean	Median	Maximum	Minimum
Ecological footprint	50674.6	50920.5	68301.3	30101.5
Physical infrastructure index	4.0	4.2	6.6	0.5
Trade openness	0.36	0.35	0.73	0.26
Urban population	41576.9	38709.3	79927.8	14429.1

Second, the prerequisite for using ARDL and NARDL model is to test the stationarity of time series data [98]. The ADF [90] and PP [91] tests examine each data series for unit root. The prerequisite for using ARDL and NARDL is to test the stationarity of time series data. The ADF [90] and PP [91] tests examine the unit root of all data series in the model. It is important to note that NARDL model employs after checking whether all data series are stationary at the level or first difference or a mixture of I (0) and I (1). However, suppose that ADF and PP suggest stationarity of any of the selected data series in the 2nd difference or I (2) model, the NARDL model is not an appropriate choice for determining the symmetrical and asymmetrical impact of explanatory variables on the ecological footprint [99]. Findings of Table 4 shows that none of the selected variables is stationary at 2^nd^ difference, which implies that the non-linear ARDL approach is applicable for this study.

**Table 4:** Results of unit root tests.

Variables	ADF test statistic			PP test Statistic		
	I(0)	I(1)	Conclusion	I(0)	I(1)	Conclusion
*log* EP	-2.29	-5.99**	I(1)	-1.64	-10.64**	I(1)
*log* II	-1.27	-6.16**	I(1)	-1.86	-20.0**	I(1)
*log*TO	-3.58**	--	I(0)	-3.65*	--	I(0)
*log*UR	-5.03**	--	I(0)	-8.34*	--	I(0)

** 5% level of Significance.

Third, this study applied the Akaike information criterion (AIC) to determine the ideal match non-linear ARDL model. The 20 best non-linear ARDL models are shown in Table 5. Fig 1 is the graphic presentation of the 20 best models based on the AIC criteria. The order of the best-fitted model is non-linear ARDL (3, 2, 1, 2, 3, 2).

**Fig 1:** Specification of the 20 best models based on AIC criteria.

**Table 5:** NARDL model specification.

Model	Log L	AIC	BIC	HQ	Adj. *R*^2^	Specification
1	109.53	-3.93	-3.18	-3.65	0.98	3,2,1,2,3,2
2	110.43	-3.93	-3.13	-3.63	0.98	3,2,1,3,3,2
3	109.41	-3.93	-3.17	-3.64	0.98	3,1,1,2,3,3
4	109.39	-3.93	-3.17	-3.64	0.98	3,0,2,2,3,3
5	114.313	-3.92	-2.97	-3.56	0.98	3,3,3,3,3,3
6	106.29	-3.92	-3.28	-3.68	0.98	3,0,2,0,3,2
7	1.28	-3.92	-3.28	-3.68	0.98	3,1,1,3,3,3
8	110.20	-3.92	-3.12	-3.62	0.98	3,0,3,2,3,2
9	109.19	-3.92	-3.16	-3.63	0.98	3,3,1,3,3,2
10	111.19	-3.92	-3.08	-3.60	0.98	3,2,1,2,3,3
11	110.18	-3.92	-3.12	-3.62	0.98	3,0,2,3,3,3
12	110.12	-3.91	-3.12	-3.62	0.98	3,1,1,2,3,2
13	108.09	-3.91	-3.20	-3.64	0.98	3,3,3,3,3,2
14	113.09	-3.91	-3.00	-3.57	0.98	3,3,1,3,3,3
15	112.08	-3.91	-3.04	-3.58	0.98	3,1,1,3,3,2
16	109.03	-3.91	-3.15	-3.63	0.98	3,0,2,2,3,2
17	108.01	-3.91	-3.19	-3.64	0.98	3,2,1,0,3,2
18	107.05	-3.91	-3.23	-3.66	0.98	3,0,3,3,3,2
19	109.95	-3.91	-3.11	-3.61	0.98	3,2,1,3,3,3
20	106.84	-3.91	-3.07	-3.59	0.98	3,0,2,0,3,3

Fourth, this study applied the F-bound test to investigate the co-integration of the data series. Table 6 shows the result of the F-bound test to explore the co-integration between the drivers of ecological footprint and ecological footprint. The F statistic value of 7.16 is more significant than the respective upper critical limit at the 1% significance level, increasing the presence of long-term asymmetric co-integration between the model’s exogenous variables and the ecological footprint in Pakistan.

**Table 6:** F-bound test results.

F-bound test statistics		
F-statistic	7.16*	
K	5	
Significance level	L_0_ (lower bound critical value)	L_1_ (upper bound critical value)
10%	2.26	3.35
5%	2.62	3.79
2.5%	2.96	4.18
1%	3.41	4.68

*1% level of significance.

Fifth, the study examined the symmetric/ asymmetric imapct of physical infrastructure and trade openness on ecological footprint using Wald test [100]. Table 7 shows the results of the symmetries test; here, the null hypothesis is that the infrastructure and trade openess in the runs are symmetric with respect to the alternative hypothesis that their imapct is asymmetric. We accept the alternative hypothesis and conclude that, both in the short run, the positive and negative partial sum of squares are significantly different from each other and support the asymmetric behavior of both infrastructure and trade openness. Furthermore, we accept the null hypothesis in the case of infrastructure and conclude that the positive and negative partial sum of squares are not significantly different from each other and support the symmetric behavior of the infrastructure in the long run. However, we accept the alternative hypothesis in the case of trade openness and conclude that the positive and negative partial sum of squares are significantly different from each other and support the asymmetric behavior of trade openness in the long run. Thus, trade openness influences the ecological footprint differently in both runs and with different levels of positive and negative effects. Meanwhile, infrastructure influences the ecological footprint asymmetrically in the short term and symmetrically in the long term. The urbanization variable cannot be transformed into an asymmetric variable due to the omission of the negative asymmetric variable [94].

**Table 7:** Test for symmetries.

Wald statistic	$X^{2}$ statistic	Prob.	Conclusion
II-SR	13.39*	< 0.01	asymmetric
TO-SR	14.12*	< 0.01	asymmetric
II-LR	0.13	0.72	symmetric
TO-LR	10.91*	< 0.01	asymmetric

*1% level of significance.

Sixth, this study employed the non-linear ARDL model to investigate the asymmetric influence of physical infrastructure and trade openness on the ecological footprint in Pakistan. Table 8 gives non-linear ARDL model turn out. The results suggest that the partial sum of positive changes in physical infrastructure is a positive factor or determinant or driver of the ecological footprint in Pakistan, both in the short and long term. This shows that a 1% increase in positive physical infrastructure shocks to zero and a lag value causes an increase of 0.34% and 0.04% in the ecological footprint in the short term, respectively. Interestingly, the partial sum of negative changes in physical infrastructure is also the main determinant of Pakistan’s ecological footprint, both in the long term and short term. A 1% reduction in the partial sum of negative physical infrastructure changes at time “t” causes a 0.02% reduction in the ecological footprint. The results also show that the partial sum of positive changes in trade openness is a positive determinant of Pakistan’s ecological footprint, both in the short and long term. The 1% increase in positive trade opening shocks in period zero and a lag period causes a 0.06% and 0.22% increase in the ecological footprint in the short term, respectively. The 1% reduction in the partial sum of negative trade openness to zero, first and second lag caused a reduction of 0.45%, 0.16% and 0.20% in ecological footprint, respectively. The results also conclude that urbanization is a significant determinant or factor of the ecological footprint in Pakistan, both in the short and long run. As the negative asymmetric variable is missig in urbanization, it cannot be turned into an asymmetric variable [94].

**Table 8:** Results of the non-linear ARDL model.

Variables	Short-run elasticities	Std. error	t-statistic	Prob.
$\Delta log{EP}_{t-1}$	0.71*	0.23	3.09	<0.01
$\Delta log{EP}_{t-2}$	0.49*	0.16	3.03	<0.01
$\Delta log{II}_{t}^{+}$	0.34*	0.10	3.33	< 0.01
$\Delta log{II}_{t-1}^{+}$	0.04	0.03	1.32	0.20
$\Delta log{II}_{t}^{-}$	0.02	0.03	0.66	0.52
$\Delta log{TO}_{t}^{+}$	0.06	0.12	0.50	0.62
$\Delta log{TO}_{t-1}^{+}$	0.22***	0.13	1.71	0.09
$\Delta log{TO}_{t}^{-}$	0.45*	0.15	3.09	< 0.01
$\Delta log{TO}_{t-1}^{-}$	0.16	0.11	1.44	0.16
$\Delta log{TO}_{t-2}^{-}$	0.20**	0.10	2.03	0.05
$\Delta log{UR}_{t}$	0.56*	0.21	2.63	< 0.01
$\Delta log{UR}_{t-1}$	0.42**	0.18	2.34	< 0.05
*ECT*_*t-1*_	-1.91*	0.30	-6.31	< 0.01
long-run elasticities				
$log{EP}_{t-1}$	-1.91*	0.30	-6.31	< 0.01
$log{II}_{t-1}^{+}$	0.32*	0.10	3.15	< 0.01
$log{II}_{t-1}^{-}$	0.33*	0.11	2.96	< 0.01
$log{TO}_{t-1}^{+}$	0.09	0.09	1.05	0.30
$log{TO}_{t-1}^{-}$	0.61*	0.18	3.50	< 0.01
$log{UR}_{t-1}$	1.31*	0.29	4.50	< 0.01
*Constant*	11.64*	4.32	2.69	<0.01

*, **, *** show level of significance at 1%, 5%, and 10%, respectively.

A 1% increase in positive shocks of physical infrastructure index causes an long run increase of 0.32% in the ecological footprint. The partial sum of negative changes in physical infrastructure is also the main determinant of Pakistan’s ecological footprint, in the long. A 1% reduction in the partial sum of negative physical infrastructure causes a 0.33% reduction in the ecological footprint. The results also show that the partial sum of positive changes in trade openness is a positive determinant of Pakistan’s ecological footprint, in the long run. The 1% increase in positive trade opening shocks causes a 0.09% increase in the ecological footprint in the long-run. The 1% reduction in the partial sum of negative trade openness caused a reduction of 0.61% in ecological footprint. The results also conclude that urbanization is a major determinant of the ecological footprint in Pakistan, in the long run. Thus, 1% increase in urbanization caused 1.31% increase in the ecological footprit in the long-run. The positive linear relationship of information and communication technology with environmental degradation is also in line with the study by Majeed [101] and Jafri, Liu [53] which is one of the important factors of the physical infrastructure of this study. Information and communication technology and roads have a linear but positive long-term correlation with the emission of CO_2_ [53]. Likewise, Asher, Garg [31] determined that transport factors are determinants of the ecological footprint. When natural systems are replaced by built infrastructure such as buildings and roads, they tend to increase the magnitude of the footprint. In addition, the physical infrastructure we use today, such as power plants, concrete roads, bridges, mines and factories, has been estimated to create a considerable amount of the environmental pollution that exists today. Furthermore, Umar, Ji [102] and Erdogan [103] consider the transport infrastructure in the long term as an important and significant factor in the emission of CO_2_. Nathaniel and Khan (2020) suggested trade as a positive determinant of the long-run ecological footprint. Likewise, Jafri et al. (2021) also confirmed the positive, long-run, but symmetrical association between trade openness and environmental degradation. In this proposed study, the emission of CO_2_ is considered as a proxy for environmental degradation, which is a large part of the contribution to the ecological footprint. Likewise, according to Erdogan (2020), trade openness is a significant and positive determinant of the ecological footprint. Rashid, Irum [104], Luo, Bai [105]; Nathaniel and Khan (2020), Nathaniel (2020), Ahmed, Zafar [62]; Hubacek, Guan [106] consider urbanization to be an important determinant of the ecological footprint, suggesting that an increase in urbanization also causes an increase in the ecological footprint. Rapid urbanization also increases the demand for non-natural resources such as electricity, water and space, which increases people’s ecological footprint and therefore has become the biggest challenge [106]. To verify the long-term stability of the non-linear ARDL model, error correction term (ECT) is introduced as cointegrating Eq (-1), which is significant at a 1% level with a negative sign. This result explains that the non-linear ARDL model is dynamically stable in the long run. It implies that 191% more imbalance adjustment would bring long-term stability to the non-linear ARDL model.

Finally, different diagnostic tests were applied to confirm whether the coefficients of the selected non-linear ARDL model are reliable, stable, and predictable or not. The results of the Breusch-Godfrey LM test [95, 96] confirmed that the specified nonlinear ARDL model is free from serial correlation problems, as the probability value of $X^{2}$ statistical is insignificant at the significance level of 5%. The results of the Ramsey’s RESET test [107] verified the normal distribution of the residual terms, as the probability value of $X^{2}$ statistical is insignificant at the significance level of 5%. The results of the Jarque-Bera test [108] verified the appropriate functional form of the model, as the probability value of F-statistical is insignificant at the significance level of 5%. In addition, CUSUM (cumulative sum of residuals) [97] and CUSUMQ (cumulative sum of squared residuals) tests [97] were used to verify the stability of the non-linear ARDL model/ parameters. The straight line represents the critical threshold at the 5% significance level. The CUSUM and CUSUMSQ statistic graphs fall into the critical regions. This confirms that the parameters of the nonlinear ARDL model are stable and reliable [97] (Fig 2A and 2B). Findings of diagnostic tests are given in Table 9.

**Fig 2:** a. Results of cumulative sum of test. b. Results cumulative sum of squares test.

**Table 9:** Findings of diagnostic tests.

Test	Type Statistic	Prob.	Conclusion
Serial correlation LM test	0.04	0.85	No serial correlation
Ramsey’s RESET test (1969)	0.90	0.35	Linear model specified correctly
Jarque-Bera (1987)	3.46	0.18	Residuals distributed normally
Cumulative sum test (1975)	-	-	Stable model/ parameters (Fig 2A)
Cumulative sum of squares test (1975)	-	-	Stable model/ parameters (Fig 2B)

## Conclusion

This study aims to explore the asymmetric impacts of physical infrastructure and trade liberalization on the ecological footprint in Pakistan, based on a non-linear ARDL model for the period 1970–2019. First, the physical infrastructure index was developed using the Principal Component Analysis (PCA) approach, including five physical infrastructure components. Second, the unit root test results show that none of the data series is stationary at the second difference, which implies that the non-linear ARDL approach is applicable for this study. Third, the order of the best fitted nonlinear ARDL is NARDL (3, 2, 1, 2, 3, 2) and was determined based on the Akaike information criterion (AIC). Fourth, the F-bound test results explored the co-integration between the factors that determine the ecological footprint. The results of the Wald test and the nonlinear ARDL model confirmed that the infrastructure influences the ecological footprint asymmetrically in the short term and symmetrically in the long term. Furthermore, trade openness influences the ecological footprint differently in both runs and with different levels of positive and negative effects. The results also conclude that urbanization is a significant factor in Pakistan’s ecological footprint, both in the short and long term. The urbanization variable cannot be transformed into an asymmetric variable due to the omission of the negative asymmetric variable. The error correction term results also concluded that the nonlinear ARDL model is dynamically stable in the long term and implies that the 191% imbalance would be adjusted in the long term. Finally, the diagnostic tests confirmed that the results of the selected nonlinear ARDL model are reliable, stable, and predictable.

Keeping in view findings of this study, policy implications are sevenfold; first, since physical infrastructure affects the ecological footprint, it is recommended that policies regarding physical infrastructure be formulated keeping in view its environmental impact. Second, trade liberalization puts pressure on the ecological footprint, it is recommended that, while stimulating its pace in Pakistan’s economy, strict environmental policies should be implemented to reduce the environmental degradation effect of trade openness. Pakistan should also participate more in market integration with its trading partners. Furthermore, environmental sustainability is a necessary condition for globalization, efforts should be made to improve the quality of the environment. Third, the results of this study also explored that urbanization increases the ecological footprint and, consequently, deteriorates environmental quality. Rural-urban migration also occurs in Pakistan due to the low standard of living and the scarcity of necessities in rural area. As a result, people migrate from rural to urban to improve their quality of life. Therefore, it is also suggested that the government of Pakistan and other stakeholders should provide basic facilities in rural areas, which will reduce rural-urban migration and lessen environmental degradation. Moreover, to achieve sustainable cities and urban area, there needs to be a reduction in population size in Pakistan. Utilizing open spaces for the creation of sustainable cities will facilitate a rapid population reduction and will reduce the pressures from both natural and social environmental factors on the consumption of limited land and resources.

Fourth, it is suggested that the Government of Pakistan needs to adopt sustainable development strategies along with environmental goals and embrace the Ecological Footprint concept to plan how they can decrease consumption of non-natural resources, physical infrastructure and transport, protecting nature and human health. It is important to identify where the gaps are in Pakistan’s environmental strategies and develop effective policies that will reduce the impact of transport and urbanization on the ecological footprint and enable sustainable economic and environmental goals. In addition, it is also recommended to introduce new economic paradigms and effective national and international institutions to achieve sustainable economic development alongside environmental sustainability.

Fifth, to lessen Pakistan’s ecological impact and improve environmental quality, it is also recommended that the country focus on improving renewable energy rather than relying solely on fossil fuels [53]. Likewise, in addition to increased investment in renewable energy, capital is needed to upgrade existing fossil power plants to improve environmental quality. Likewise, the green bank is an environmental strategy that aims to increase funding for clean energy projects to improve environmental quality and reduce the environmental footprint. However, in Pakistan, government and academics are struggling to establish economic policies to invest in green industry and reduce carbon emissions [109]. Green Banking or investment banking to increase green production to decrease the environmental footprint and reduce CO_2_ emissions to a certain level is crucially suggested. Moreover, as public development expenditures has positive association with ecological footprint in Pakistan [13], therefore, a viable and concrete fiscal policy is recommended, especially in the sphere of infrastructure development, which can enable Pakistan to achieve the SDGs (Sustainable Development Goals).

Sixth, in the process of controlling environmental degradation, the asymmetric role of trade liberalization and physical infrastructure in the ecological footprint must be played out to help the Government of Pakistan determine goals for sustainable economic development. In the process, it will be learned which ecological footprint determinants are causing economic growth to decline and what steps need to be taken to reverse this trend. Therefore, the term ecological footprint describes a set of behaviors that must be changed if we want our planet to survive the next century.

Seventh, it is important to note that this study investigates the non-linear impact of physical infrastructure, including only a few determinants in the index, although there are many other determinants of physical infrastructure that may have their influence on the ecological footprint in Pakistan, such as power grids, waste grids. and sewage system. Likewise, the specific infrastructure used for trade can also impact as a trade opening factor in the ecological footprint that is not included in the study. These two are the main limitations of this study. The existing study paved the way for including the wide variety of physical infrastructure factors in the index to further pinpoint these results for a more detailed perspective.
